The article "Upregulated expression of long non-coding RNA MEG3 serves as a prognostic biomarker in severe pneumonia children and its regulatory mechanism" was published in 2021. Journal: Bioengineered.

# Upregulated expression of long non-coding RNA MEG3 serves as a prognostic biomarker in severe pneumonia children and its regulatory mechanism

**DOI:** 10.1080/21655979.2021.1979351

**Published:** 2021-09-24

**Authors:** Jie Guo, Ning Zhang, Guozhi Liu, Aimei Zhang, Xin Liu, Jie Zheng

**Affiliations:** a Department of Neonatology, Yidu Central Hospital of Weifang, Weifang, Shandong, 262500, China; b Department of Neonatology, Weifang People’s Hospital, Weifang, Shandong, 261041, China

**Keywords:** MEG3, miR-29c, prognosis, diagnosis, inflammation, viability

## Abstract

Severe pneumonia is a high-mortality disorder in children. The expression and underlying effects of lncRNA maternally expressed 3 (MEG3) were detected. The relationships between MEG3 and other parameters were reported by Pearson correlation. The prognostic importance of MEG3 was assessed by Kaplan-Meier (K-M) curve and COX analysis and its diagnostic potential was uncovered by the receiver operating characteristic (ROC) curve. Luciferase activity assay was performed to demonstrate the target gene of MEG3. Elevated expression of MEG3 and reduced microRNA-29 c (miR-29 c) were evaluated in severe pneumonia children, and a negative relationship between MEG3 and miR-29 c was propounded. MEG3 might function as an independent prognostic indicator. The diagnostic efficiency of MEG3 was also indicated for severe pneumonia children. In MRC-5 cell models and MH-S cell models, lipopolysaccharide (LPS) contributed to the increased expression of MEG3. Interference of MEG3 restricted the upregulation of MEG3 triggered by LPS. Silenced MEG3 protected MRC-5 and MH-S cells against damages managed by LPS on cell apoptosis, viability, and inflammation. MiR-29 c was a ceRNA of MEG3 and the absence of MEG3 abrogated the decreased expression of miR-29 c caused by LPS. Overall, the increased expression of MEG3 and the reduced levels of miR-29 c were identified in severe pneumonia. Prognostic and diagnostic significances of MEG3 provided a novel perspective for severe pneumonia. Disruption of MEG3 alleviated cell injury and inflammation as characterized by high LPS by binding miR-29 c.

## Background

Pneumonia is a pulmonary tissue inflammatory disorder, which usually infects children [1,2]. Despite the effective prevention through vaccination, pneumonia is still perceived as a leading death threat to children [3]. According to an investigation about disease burden, approximately 14% of children die of pneumonia globally [4]. Severe pneumonia is accompanied by complex clinical manifestations, like hypoxemia, dyspnea, elevated body temperature, mental status changes, hypotension, or other severe comorbidities [5]. Currently, radiological technology and multiple laboratory methods are the main diagnostic methods, whereas, the clinical impact of radiology needs to be further determined, and laboratory examination lacks accuracy in host differentiation [6]. Accordingly, the timely diagnosis and accurate prognosis of severe pneumonia are paramount in clinical management.

Long non-coding RNA (lncRNA) regulates the progression of disorders or biological activities by binding target genes or microRNAs (miRNAs). Tissue-specific and condition-specific expression characters of lncRNAs suggest that they are potential biomarkers and provide a rationale to apply them clinically [7]. Enormous researches focused on the fundamental significance of lncRNAs and pneumonia are published and these studies contribute to the clinical management of pneumonia patients and the mechanism underlying pneumonia. In an investigation of elderly patients with severe pneumonia, lncRNA MALAT1 may function as a biomarker for the prognosis, which opens up new insights on predicting pneumonia [8]. Consistently, a publication about acute pneumonia not only identifies the highly expressed levels of lncSNHG16 in patients with acute pneumonia but also explains the underlying causes, namely silenced SNHG16 facilitates cell viability and suppresses cell apoptosis by sponging miR-146a-5p [9]. LncRNA maternally expressed 3 (MEG3) exists in several tissues and interacts with different genes or miRNAs, which further plays roles in diseases’ intervention or treatment, including pulmonary lesions or relevant disorders [10]. Aberrant expression of MEG3 modulates the amount of Th17 and influences Treg/Th17 balance in asthma by combining miRNA-17 [11]. Besides, MEG3 alters the proliferation and invasion of lung cancer cells and plays as a promising target in lung cancer [12]. In a previous publication, MEG3 is also expressed at higher levels in epithelial cells separated from patients with idiopathic pulmonary fibrosis [13]. Nevertheless, the expression of MEG3 in severe pneumonia children as well as its possible application and mechanism are elusive.

MEG3 might play roles in the clinical management of severe pneumonia. To test this hypothesis, this current experiment aimed to detect the expression of MEG3 in severe pneumonia children and its association with clinical characteristics. For the clinical management, the prognostic significance and diagnostic accuracy of MEG3 were evaluated. Additionally, the molecular mechanism of MEG3 relative to the pathogenesis of severe pneumonia was investigated.

## Methods

### Patients and sample collection

A total of 77 healthy children and 88 children with severe pneumonia were recruited in this investigation from Weifang People’s Hospital. The diagnosis strictly followed the criteria of clinical management guidelines of the American Infectious Diseases Association [14]. The major criteria were respiratory failure, which needs noninvasive positive pressure or invasive ventilation and septic shock occurs. Some other minor criteria were also conducted, such as respiratory rate, oxygenation index, or blood pressure. Once the patient had one of the aforementioned major symptoms or three of minor criteria, he or she was diagnosed with severe pneumonia patients. In 88 patients with severe pneumonia, there were 56 positive cases, including 32 bacterial infections, 11 virus infections, 4 fungal infections, 6 mycoplasma infections, and 3 chlamydia infections. All children received routine symptomatic treatment, including vital signs monitoring, nutritional support, oxygen inhalation, and antibiotics. Patients with preexisting diseases, including congenital malformation and immunodeficiency, were limited to this study. All these patients received a 28-day follow-up and the survival outcome of each patient was summarized. The vein blood samples were isolated from patients within 12-hours of diagnosis. The healthy individuals were chosen randomly from the pediatric department of the same hospital. Patients with chronic infectious or immune disease, malignancy, allergy, or intimate contact with infectious victims were restricted from inclusion in this study. The plasma specimens were collected after centrifuging blood samples.

This study was approved by the Weifang People’s Hospital ethics committee and written informed consent was collected from legal guardians of included patients. All protocols were performed as per the Declaration of Helsinki.

### RNA extraction and quantitative real-time PCR (qRT-PCR)

RNA samples were extracted from plasma specimens using TRIzol reagent (Invitrogen, Carlsbad, USA). Regarding miR-29 c, the first line of complementary DNA (cDNA) was synthesized by a reverse transcription kit (Applied Biosystems, Foster City, USA). One Tube RT-PCR kit (Roche, Basel, Switzerland) was applied to obtain cDNA of MEG3. FastFire qPCR PreMix (SYBR Green) (TIANGEN, Beijing, China) was purchased to evaluate the relative expression in MRC-5 cells, MH-S cells, and patients. U6 and β-actin served as normalized reference genes and the 2^−ΔΔCt^ method was used to calculate expression based on the data of the ABI 7300 system (Applied Biosystems, Foster City, USA).

### Cell cultivation and model construction

Human lung fibroblast cells MRC-5 were obtained from EK-Bioscience (Shanghai, China) and fostered in MEM supplemented with 1% compound antibiotic and 10% FBS at 37°C in an incubator full of 95% air and 5% CO_2_. Different concentrations of lipopolysaccharide (LPS) (0 μg/ml, 5 μg/ml, 10 μg/ml, 20 μg/ml) were separately mixed into medium to mimic injured cell condition after 24-hour incubation [15]. LPS (Escherichia coli serotype 055:B5) from Sigma-Aldrich (St. Louis, USA) was used in our experiment. Besides, murine alveolar macrophages (MH-S) cell lines were obtained from Procell company (Wuhan, China) and fostered in RPMI-1640 medium with 10% at 37°C. LPS (1 μg/ml) was used to treat MH-S cells for 24 hours to established LPS-injured cell models [16].

### Gene transfection

Sangon (Shanghai, China) was entrusted to synthesize si-MEG3 and its negative controls (si-NCs) together with miR-29 c mimics, miR-29 c inhibitors, and miR-NCs. The transfection experiments were implemented using lipofectamine 3000 (Life Technologies, Carlsbad, USA) in line with the recommended instruction.

### In vitro assay

For detection of cell viability, Cell Counting Kit-8 (CCK-8) was applied to this experiment [17]. Experimental cell suspension was seeded into a 96-well plate. The density was 5 × 10^3^ cells/well. After being fostered for 24 hours, 10 μl Cell Counting Kit-8 (CCK-8) reagent (Dojindo, Kumamoto, Japan) was added to the cell suspension. The absorbance at 450 nm was obtained using a microplate reader (Molecular devices, CA, USA).

Flow cytometry was used to analyze the cell apoptosis. Experimental cells were gathered and washed by PBS. About 5 × 10^5^ cells were suspended by 500 μl binding buffer. Then, 5 μl Annexin V-EGFP and 5 μl Propidium Iodide were mixed with cell suspension. Subsequently, cells were stained for 30 minutes in dark. A flow cytometry (Beckman, Fullerton, CA) was utilized to assess cells. The reagents utilized in this assay were from Annexin V-EGFP Apoptosis Detection Kit (Keygen Bio, Nanjing, China) [18].

### Enzyme-linked immunosorbent assay (ELISA)

The culture supernatant of MRC-5 cells and MH-S cells was collected after incubation with LPS. ELISA kits (R&D Systems, Minneapolis, USA) were utilized to the concentration of TNF-α, IL-6, and IL-1β [19].

### Luciferase activity assay

Wide type (WT)-MEG3 containing binding sites were amplified by PCR using Ultra HiFidelity PCR Kit (TIANGEN, Beijing, China), and mutation type (MUT)-MEG3 was synthesized by Sangon (Shanghai, China). The obtained MUT-MEG3 and WT-MEG3 sequences were cloned into pmirGLO vectors. The vectors carried with WT-MEG3 were co-transfected with miR-29 c mimics, miR-29 c inhibitors, or miR-NC into MRC-5 cells via lipofectamine 3000 ((Life Technologies, Carlsbad, USA). The co-transfection procedures of MUT-MEG3 were consistent with that of the WT-MEG3 group. Luciferase activities were surveyed 48 hours after transfection utilizing the Dual-Glo luciferase system kit (Promega, Madison, USA) [20].

### Statistical analysis

The exhibited consequences were calculated via SPSS 19.0 and GraphPad 5.0. All experiments were implemented independently in triplicate. The significances of different groups were accessed by T-test, chi-square test, and one-way analysis of variance. The correlation between MEG3 and miR-29 c was analyzed with Pearson correlation. Clinical values of MEG3 were dealt with Kaplan-Meier (K-M) test, the log-rank test, together with the receiver operating characteristic (ROC) curve and Cox regression test.

## Results

Our study aimed to evaluate the clinical implication and potential mechanism of MEG3 in severe pneumonia. For this purpose, we explored the diagnostic value and prognostic accuracy of MEG3 for severe pneumonia children. Besides, the effects of MEG3 on the viability, apoptosis, and inflammation of MRC-5 cells and MH-S cells were investigated. Furthermore, the mechanism underlying MEG3 was also explored.

### Baseline clinicopathological manifestation

The clinical data were recorded and expressed in Table 1. The severe pneumonia group was constituted of 56 males and 32 females with an average age of 6.25 ± 1.53 years old. There were no significant differences in the gender, age, and body mass index (BMI) between severe pneumonia patients and healthy children, suggesting the two groups have statistical comparability (*P* > 0.05, Table 1). Some laboratory items, such as the white blood cell (WBC) count and lymphocytes, showed no statistical significance between severe pneumonia patients and healthy children (*P* > 0.05, Table 1). In addition, neutrophils, C-reactive protein (CRP), lactate dehydrogenase, and procalcitonin (PCT) were significantly higher in the severe pneumonia group than those in control children (*P* < 0.001, Table 1). These conclusions of clinical items implied the obvious damage and severe inflammatory response contributed by severe pneumonia. Besides, 34 patients were delayed for at least 5 days from symptom onset to hospital admission, and other patients were in hospital within 5 days after symptom onset (Table 1).

**Table 1:** Clinical data of the subject population

Parameter	Healthy individuals (n=77)	Severe pneumonia (n=88)	*P*-value
Gender (male/female)	40/37	56/32	0.129
Age	5.97±1.69	6.25±1.53	0.274
BMI	22.01±2.4	22.22±2.12	0.546
WBC (10^9^**/**L)	9.71±1.71	10.20±2.17	0.114
Neutrophils	3.84±1.12	15.38±3.05	<0.001
CRP (mg/L)	3.45±1.35	12.80±1.68	<0.001
Lactate dehydrogenase (U/L)	240.71±43.48	301.68±86.80	<0.001
Lymphocyte (10^9^**/**L)	2.56±0.61	3.00±2.13	0.084
PCT (ng/mL)	0.14±0.07	2.05±0.80	<0.001
Delay from symptom onset to hospital admission			
≥5 days	-	34	-
<5 days	-	54	-

Note: BMI, body mass index; WBC, white blood cell; CRP, C-reactive protein; PCT, procalcitonin; data are expressed as n or mean ± standard deviation.

### High levels of MEG3 in patients

The prominent enhancement of MEG3 expression was verified in the severe pneumonia group in comparison with the expression of MEG3 in healthy groups, which propounded severe pneumonia might contribute to the obvious abundance of MEG3 expression (*P* < 0.001, Figure 1a).

**Figure 1.** The expression and clinical significance of MEG3. **A** High level of MEG3 was identified in children with severe pneumonia. **B** ROC result indicated the predictive significance of MEG3. **C** Increased levels of MEG3 contributed to a worse survival outcome. ***P < 0.001

### Clinical values of MEG3 for severe pneumonia patients

The ROC result showed the predictive value of MEG3 in severe pneumonia, which was exhibited in Figure 1b. The finding demonstrated the area under the curve (AUC) was 0.922, indicating the possibility of MEG3 as a satisfactory diagnostic marker. Also, the sensitivity (80.7%) and specificity (89.6%) were propounded the superiority of MEG3 in severe pneumonia.

Further analysis was put into practice to redouble the correlation between MEG3 and various markers in severe pneumonia. As elucidated in Table 2, no correlations were found between MEG3 expression and age, BMI, WBC, lymphocyte, and delay from symptom onset to hospital admission (*P* > 0.05). MEG3 was weakly correlated with the degree of lactate dehydrogenase (R = 0.299, *P* = 0.005, Table 2). Significantly, there were close linear correlations between MEG3 and neutrophils (R = 0.772, *P* < 0.001, Table 2), CRP (R = 0.634, *P* < 0.001, Table 2), and PCT (R = 0.727, *P* < 0.001, Table 2), highlighting that MEG3 had a high possibility as a promising biomarker in severe pneumonia.

**Table 2:** Correlation between MEG3 and various indicators

Paraments	Correlation with MEG3 (r)	*P-value*
Age	0.036	0.742
BMI	0.158	0.141
WBC (10^9^**/**L)	0.159	0.069
Neutrophils	0.772	<0.001
CRP (mg/L)	0.634	<0.001
Lactate dehydrogenase (U/L)	0.299	0.005
Lymphocyte (10^9^**/**L)	0.058	0.594
PCT (ng/mL)	0.727	<0.001
Delay from symptom onset to hospital admission	0.145	0.177

Abbreviations: BMI, body mass index; WBC, white blood cell; CRP, C-reactive protein; PCT, procalcitonin.

### MEG3 indicated the suboptimal outcome of severe pneumonia patients

Based on the average expression levels of MEG3, total patients were divided into a high-level group and a low-level group. As elucidated in Figure 1c, the patients in the low-level group manifested a significantly lower overall survival percentage than that in the low-level group, providing patients with high expression of MEG3 had a worse survival outcome (*P* = 0.025). More importantly, the Cox data further underlined this finding, which demonstrated MEG3 (HR = 2.981, 95%CI = 1.159–7.664, *P* = 0.023), PCT (HR = 2.574, 95%CI = 1.029–6.434, *P* = 0.043), and delay from symptom onset to hospital admission (HR = 2.522, 95%CI = 1.080–5.887, *P* = 0.032) were alternative independent biomarkers for predicting overall survival of patients with severe pneumonia (Table 3).

**Table 3:** Multivariate Cox analysis of clinical characteristics in relation to overall survival

Characteristics	Multivariate analysis		
	HR	95% CI	*P*
Lnc MEG3	2.981	1.159 – 7.664	0.023
Gender	1.531	0.635 – 3.690	0.342
Age	1.225	0.510 – 2.944	0.649
BMI	0.491	0.202 – 1.191	0.115
WBC	0.558	0.239 – 1.300	0.176
Neutrophils	0.904	0.360 – 2.272	0.831
CRP	0.423	0.176 – 1.014	0.054
Lactate dehydrogenase	1.079	0.455 – 2.559	0.862
Lymphocyte	1.130	0.475 – 2.6848	0.783
PCT	2.574	1.029 – 6.434	0.043
Delay from symptom onset to hospital admission	2.522	1.080 – 5.887	0.032

Abbreviations: BMI, body mass index; WBC, white blood cell; CRP, C-reactive protein; PCT, procalcitonin.

### Influence of MEG3 on cell models

An LPS concentration gradient was added to construct the injured MRC-5 models and mimic lung fibroblast cell conditions in severe pneumonia patients. As shown in Figure 2a, cell viability was obviously decreased with the increasing LPS concentration, indicating cell models were successfully established (*P* < 0.05). On the contrary, the expression of MEG3 was varied directly as the incremental LPS (*P* < 0.05, Figure 2b). As one of the most significant differences, 10 μg/ml LPS was determined to apply in the following cell experiments with the consideration of LPS impact and virulence.The expression of MEG3 was significantly increased in the LPS group and si-MEG3 transfection successfully reversed the elevated trend of MEG3 (*P* < 0.01, Figure 2c). The viable cells were conspicuously reduced in the LPS as the previous finding, while the knockdown MEG3 obviously restored the weak cell viability (*P* < 0.01, Figure 2d). LPS contributed to the apoptosis in the MRC-5 cells, however, interfered MEG3 apparently mitigated the damage stimulated by LPS (*P* < 0.001, Figure 2e). The inflammatory actions were remarkably ascended in LPS-engendered MRC-5 cells, and the absence of MEG3 hindered this injury partly by attenuating the levels of TNF-α, IL-6, and IL-1β (*P* < 0.001, figure 2f).

**Figure 2.** The effects of MEG3 on MRC-5 cell model. **A** Increased LPS concentration led to gradually decreased cell viability. **B** The expression of MEG3 was elevated with the increased LPS dosage. **C** Transfection experiments successfully inhibited the levels of MEG3. **D-F** The influence of MEG3 on cell viability, apoptosis, and inflammation. *P < 0.05, **P < 0.01, ***P < 0.001, compared to control; ##*P* < 0.01, ###*P* < 0.001, compared to LPS group

Additionally, in the MH-S cells, the MEG3 expression was enhanced in the LPS group and si-MEG3 inhibited the expression of MEG3 significantly (*P* < 0.001, Figure 3a). The damages on cell viability, cell apoptosis, and inflammation induced by LPS were reversed partly by the reduced MEG3 expression (*P* < 0.001, Figure 3b-d).

**Figure 3.** The influence of MEG3 on MH-S cell model. **A** LPS elevated the expression of MEG3 and si-MEG3 decreased the MEG3 expression. **B-D** Absence of MEG3 protected MH-S cells against the damage of LPS on viability, apoptosis, and inflammation. ***P < 0.001, compared to control; ###*P* < 0.001, compared to LPS group

### MEG3 was a ceRNA of miR-29 c

The putative target sequence between MEG3 and miR-29 c was elucidated in Figure 4a. Besides, luciferase assay substantiated this deduction by the conclusion that upregulation of miR-29 c restricted luciferase activity, and raised activity was induced by the downregulation of MEG3 (*P* < 0.001, Figure 4b). Interestingly, miR-29 c was at low levels in LPS cell models and inhibition of MEG3 meliorated the expression of miR-29 c, further accentuating the inverse concentration relationship between MEG3 and miR-29 c (*P* < 0.01, Figure 4c). Besides, the relative expression of miR-29 c was lower in the severe pneumonia group than that in control individuals (*P* < 0.001, Figure 4d). Moreover, there was a distinct negative proportionate between MEG3 and miR-29 c in patients with severe pneumonia (R = −0.797, *P* < 0.001, Figure 4e).

**Figure 4.** MiR-29 c was a target of MEG3. **A** The probable binding bases between MEG3 and miR-29 c. **B** The exhibition of luciferase assay. **C** In the MRC-5 and MH-S cells, the expression of miR-29 c was declined in the LPS group and raised in the LPS+si-MEG3 group. **D** Decreased miR-29 c was found in severe pneumonia children. **E** Negative correlation between MEG3 and miR-29 c. **P < 0.01, ***P < 0.001

### MiR-29 c mediated the impacts of MEG3

To study whether MEG3 regulated LPS-stimulated cell injury was mediated by miR-29 c, MRC-5 cells and MH-S cells were co-transfected with si-MEG3 and miR-29 c inhibitors. In MRC-5 cells, silenced MEG3 elevated the expression of miR-29 c, while co-transfection of si-MEG3 and miR-29 c inhibitors inhibited the overexpression of miR-29 c (*P* < 0.001, Figure 5a). In addition, the intervention of miR-29 c reversed the function of MEG3 on cell viability, apoptosis, and inflammatory situation (*P* < 0.001, Figure 5b-d). The analysis of MH-S cells found that the expression of miR-29 c was raised in the si-MEG3 group and lessened in the si-MEG3+ miR-29 c inhibitor group (*P* < 0.05, Figure 6a). Besides, miR-29 c could mediate the impacts of MEG3 on the aspects of cell viability, apoptosis, and inflammation (*P* < 0.001, Figure 6b-d).

**Figure 5.** The mediated function of miR-29 c in MRC-5 cells. **A** The expression of miR-29 c was elevated in the si-MEG3 group and inhibited in the si-MEG3+ miR-29 c inhibitor group. **B-D** MiR-29 c mediated the function of MEG3 on cell viability, apoptosis, and inflammation. ***P < 0.001, compared to LPS; ###*P* < 0.001, compared to si-MEG3 group

**Figure 6.** The mediated function of miR-29 c in MH-S cells. **A** The expression of miR-29 c was elevated in the si-MEG3 group and inhibited in the si-MEG3+ miR-29 c inhibitor group. **B-D** The effects of MEG3 on cell viability, apoptosis, and inflammation were reversed by miR-29 c. **P < 0.01, ***P < 0.001, compared to LPS; #*P* < 0.05, ###*P* < 0.001, compared to si-MEG3 group

## Discussion

As a lower respiratory tract infection, the overall hospitalization rate of pneumonia is high [21]. Pneumonia is usually caused by bacteria and viruses, which is a leading disorder leading to the death of children [22,23]. Pneumonia accounts for the highest proportion of children globally, and 20% of patients need intensive care [1]. Severe pneumonia weakens the immune system, which finally leads to respiratory system injury, multiple organ failure, and even stock [24]. Modern management including empiric antibiotics and adjunctive therapies has been adopted to prevent the course of pneumonia, but complicated otherness influences therapeutic effect [25]. LncRNAs have been explored by a great number of authors, especially in pneumonia. Profiling of sequencing technique determines 99 aberrant expressed lncRNA in mild pneumonia patients and 85 dysregulated lncRNAs in patients with severe pneumonia [26]. Overexpression of lncRNA UCA1 is identified in LPS-induced cell models and it is involved in the regulation of cells by combining the miR-499b-5p/UCA1 axis [27]. Collectively, observations of lncRNAs in severe pneumonia provide conceivable perspectives for the potential mechanism of severe pneumonia.

In this study, the raised expression of MEG3 was determined in severe pneumonia patients, implying the anomalously expressed MEG3 might modulate the course of pneumonia. In a publication, MEG3 is abundant in idiopathic pulmonary fibrosis and plays as a mediator in the development of this lung disorder [13]. In a study about chronic obstructive pulmonary disease, MEG3 is at a high level in lung tissues of patients, which is coincident with our findings [28]. Our experiment of ROC provided a high sensibility and specificity of MEG3, indicating that MEG3 might be applied as a diagnostic biomarker for discriminating severe pneumonia occurrence. Currently, CRP and PCT were explored for their clinical values in the management of pneumonia, but their utilization was challenged due to the accuracy [29]. By comparison, MEG3 might be an alternative biomarker for patients with severe pneumonia. In a noteworthy investigation of severe pneumonia, MALAT1 has a prognostic value in elderly patients [8]. Besides, the elevated expression of NNT-AS1 is proportionate to CRP and PCT in children with refractory pneumonia, and NNT-AS1 may distinguish these patients with high accuracy [30]. More importantly, the correlation findings documented the levels of MEG3 were closely associated with neutrophils, CRP, and PCT, punctuating the clinical significance of MEG3 in severe pneumonia. Subsequently, the K-M curve propounded a worse overall survival in group with high MEG3 expression than in low MEG3 level group and this result was further verified by the analysis of multivariate Cox, which indicated MEG3 could serve as a promising marker in severe pneumonia independently. However, the utilization of MEG3 for patients with severe pneumonia still needs more studies.

Emerging pieces of evidence on the pathophysiology of non-coding RNAs in infectious diseases have been published recently [31]. For instance, elimination of MIAT suppressed cell apoptosis, and ultimately protect the balance of lung function via miR-147a/NKAP crosstalk [32]. Besides, SNHG16 partially restores the damage of LPS in A549 cells on the aspects of cell viability, inflammation, and apoptosis [33] Interference of circ-0059930 can notably improve proliferation and inhibit apoptosis of LPS-induced MRC-5 cells [34]. In the in vitro investigations, MEG3 was overexpressed with the increased LPS concentration and the interference of MEG3 reversed the upregulation of MEG3. Furthermore, LPS attenuated cell viability and exaggerated cell apoptosis in MRC-5 and MH-S cells, whereas, disruption of MEG3 abrogated these adverse influences, uncovering the protective roles of silenced MEG3. Additionally, knockdown of MEG3 mitigated inflammatory damage in the MRC-5 and the MH-S cell models triggered by LPS. Based on several projects, MEG3 fortifies the inflammatory cytokines and manages cell function remarkably [35,36]. A currently published study explores LPS contributed to the upregulation of MEG3 and MEG3 enhanced cell inflammation [37]. Taken together, low levels of MEG3 might function as a protective regulated in ameliorating cell injury and inflammation.

In the aspects of the regulatory mechanism of MEG3, miR-29 c was a sponge of MEG3. A previous investigation indicates MEG3 modulates cell proliferation by sponging miR-29 c in meningioma, pinpointing the regulatory relationship between MEG3 and miR-29 c again [38]. Lessened miR-29 c was found in the patients with severe pneumonia and LPS-steered cell models. In mycoplasma pneumonia, the levels of miR-29 c are declined in the children suffering from this pneumonia [39]. Further Pearson analysis result provided the expression of MEG3 was inversely associated with the levels of miR-29 c, which emphasizing MEG3 was a ceRNA of miR-29 c. More importantly, miR-29 c could mediate the function of MEG3 on cell viability, apoptosis, and inflammation. One limitation of this study was the exclusion of a group of children with mild pneumonia. Besides, the lack of the impacts of MEG3 on nuclear factor-kappa B (NF-kB) also limited this study.

## Conclusions

To sum up, MEG3 was significantly overexpressed, whereas miR-29 c was at a lower level both in severe pneumonia children and LPS-irritated MRC-5 and MH-S cell models. The expression of MEG3 was inversely associated with the amount of miR-29 c, and MEG3 might be a sponge of miR-29 c. Obvious high expression of MEG3 led to a worse outcome, and it might serve as an independent biomarker. Abnormal alteration of MEG3 could prominently discriminate severe pneumonia patients from healthy children. Elimination of MEG3 might be a protective agent, which could distinctly ameliorate cell viability, hinder cell apoptosis, and inhibit cell inflammation by sponging miR-29 c.

## Highlights

1. LncRNA MEG3 was ascended in patients with severe pneumonia.

2. LncRNA MEG3 could be a diagnostic and prognostic biomarker.

3. LncRNA MEG3 might regulate the injury induced by LPS via sponging miR-29c.
